The article "Lambert-Eaton Myasthenic Syndrome in Lung Cancer" was published in 2022. Journal: Contrast Media Mol Imaging.

# Lambert-Eaton Myasthenic Syndrome in Lung Cancer

**DOI:** 10.1155/2022/3912376

**Published:** 2022-07-05

**Authors:** Yongbin Wang, Chuanguo Xu, Yu Wang, Feifei Feng, Hui Wang, Ying Zhang, Xiaojuan Lin, Bin Xu

**Affiliations:** ^1^Department of Respiratory Medicine, The Second Hospital of Shandong University, Jinan, Shandong 250033, China; ^2^Department of Anesthesiology, Tai'an Maternity and Child Care Hospital, Tai'an, Shandong 27100, China; ^3^Department of Neurology, Fujian Geriatric Hospital, Fuzhou 350003, China

## Abstract

The aim is to study lung cancer with Lambert-Eaton myasthenic syndrome (LEMS) with clinical and electrical characteristics of physiology and prognosis. Fourteen LEMS patients with lung cancer were studied retrospectively. The data including demographics, clinical presentation, treatments, and prognosis from the medical records were analyzed. Lung cancer coexisting with LEMS is more common in men (10/14). The median age was 67.1 years. Eleven (78.6%) patients experienced gradual onset of disease. Most patients presented nervous system lesions prior to occult tumors. The most common symptoms reported were proximal muscle weakness (92.9%), decreased or absent tendon reflexes (50%), and autonomic dysfunction (71.4%). All the patients showed reduction in action potential amplitude after repetitive peripheral never stimulation at low frequency and increased amplitude at high frequency. LEMS usually occurs prior to lung cancer with complicated and various clinical manifestations in our centers. We should improve awareness and knowledge of such disease to shorten the diagnostic delay and lead to few misdiagnoses.

## 1. Introduction

Lambert-Eaton myasthenic syndrome (LEMS) is an autoimmune neuromuscular disorder that affects the presynaptic neuromuscular junctions [1]. LEMS is a rare disease with an estimated worldwide prevalence of around 1/250,000–1/333,300 previously [2]. The exact incidence of LEMS in China is unknown. Nearly half of subjects with LEMS have an associated tumour. LEMS was first recognized clinically in association with lung cancer [3]. Approximately 50 to 75% of subjects with LEMS have lung cancer, especially small cell lung cancer (SCLC) [1]. The incidence of SCLC combined with LEMS was estimated to be approximately 3% [1–4]. Given that SCLC accounts for 14% of all newly diagnosed cases of lung cancer, the number of LEMS patients with lung cancer was large, which should not be ignored [5].

Data concerning LEMS in lung cancer has been mainly obtained from case reports or small series from New Zealand, Europe, and America [6–9]. Our knowledge of the clinical and pathological features of LEMS coexisting with lung cancer was limited, especially in China. We should improve awareness and knowledge of such disease to shorten the diagnostic delay and lead to fewer misdiagnosis. Hence, we evaluated the clinical characteristics, treatments, and prognosis in lung cancer patients coexisting with LEMS in order to enhance further understanding with regard to the diagnosis and treatment.

## 2. Methods

### 2.1. Design and Measures

We conducted this study to review the patient database of Fujian Geriatric Hospital and the Second Hospital of Shandong University from 2013 to 2020 and to evaluate and analyze the subjects with lung cancer coexisting with LEMS. We reviewed the structured checklist and their clinical records to collect data. Data were collected including age, gender, date of appearance of symptoms, time to diagnosis, clinical presentation, treatments, and prognosis. The study was approved by the Ethics committee of Fujian Geriatric Hospital and the First Affiliated Hospital of Fujian Medical University. The study was conducted in accordance with the Declaration of Helsinki (as revised in 2013). No informed consent was required due to the retrospective nature of the study. Patient information was anonymized and identified prior to analysis.

### 2.2. Definition

Diagnostic criteria for LEMS in our centers are based on characteristic clinical features (proximal muscle weakness, autonomic dysfunction, and reduced or absent tendon reflexes), electromyographic features, and immunological testing (anti-VGCC antibody assay). Electromyographic features were detected by means of an electromyograph (EMG, low amplitude of the compound muscle action potential and increment after high-frequency stimulation or maximal voluntary contraction). Staging of lung cancer in all study patients was classified by the more recent tumor, node, metastasis (TNM) staging (stage I to IV) from the International Association for the Study of Lung Cancer. Acute-onset could be defined as symptoms onset less than 2 weeks. Gradual-onset could be defined as symptoms onset more than 2 weeks.

### 2.3. Statistical Analysis

We performed statistical analysis using Statistical Product and Service Solutions (SPSS) software for Windows, version 21.0 (IBM, Armonk, NY, USA). Descriptive summary of demographic, clinical variables, and other data was performed for continuous variables as mean ± standard deviation (SD) or median (interquartile range) as appropriate and categorical variables as frequency percentages.

## 3. Results

Our retrospective analysis identified 14 patients with the LEMS associated with lung cancer. Demographic and clinical variables are presented in Table 1. Of these cases, 9 patients were male, and 5 patients were female (1.8 : 1). Median age at diagnosis was 61.3 ± 12.7 years. Three patients had smoking history (21.4%), and ten patients (71.4%) are current smokers. Thirteen patients (92.9%) developed SCLC, while only one patient developed lung adenocarcinoma. Nine (64.3%) patients had stage III-IV. Nine (64.3%) patients had good performance status score of 0 or 1 at baseline. All patients were evaluated or managed by neurologists and pulmonary physicians. Ten patients received voltage-gated calcium channel (VGCC) antibodies test. Positive results for VGCC antibodies were found in 7 patients. Onset of LEMS preceded lung cancer diagnosis in 12 cases (85.7%) and was concurrent in 2 patients (14.3%). Median time between diagnosis of LEMS and detection of the lung cancer in these 12 patients was 5 months (range, 0.5 to 15 months). The median interval between onset of symptoms and complete diagnosis of lung cancer coexisting with LEMS was 11.9 months. The longest delay diagnosis between onset and final diagnosis was 3 years. Initially, 12 patients (85.7%) were misdiagnosed with other diseases, including peripheral neuropathy (*n* = 10), myasthenia gravis (*n* = 1), motor neuron disease (*n* = 1), lower body parkinsonism (*n* = 1), and lacunar infarction (*n* = 1). Three cases had a concurrent immunological disorder including rheumatoid arthritis (*n* = 2) and systemic vasculitis (*n* = 1).

In most patients, the onset was gradual (78.6%), but only three cases were acute (21.4%). Early symptoms of six patients presented without respiratory symptoms and/or signs. The chest CT scan was found to be abnormal in all patients. The frequencies of symptoms and signs were analyzed (Table 2). Patients had developed on average four separate neurologic symptoms and signs. Most common presenting symptoms or signs were proximal leg weakness (60%), followed by dry mouth (57.1%) and decreased or absent tendon reflexes (50%). The frequency of ocular and bulbar symptoms was 21.4% and 28.6%, respectively. Symptoms or signs of autonomic dysfunction were found in 71.4% of patients. Dry mouth (57.1%) and constipation (42.9%) was probably the common symptoms of autonomic dysfunction. Three patients developed respiratory muscle weakness requiring noninvasive ventilation. They were either misdiagnosed or not treated for LEMS at the time of perioperative complication and developed hypoxemia after using neuromuscular blocking drugs. Seven patients (50%) showed decreased or absent tendon reflexes.

Respiratory abnormalities on spirometry were found in six patients. Three patients had mild to moderate restrictive ventilatory dysfunction. All patients had abnormal decremental responses with low-rate stimulation and incremental responses with high-rate stimulation. No more neurons and myogenic damage were observed in all patients.

Follow-up duration ranged from 6 months to 5 years. All patients received cancer therapeutics. Initial chemotherapeutic regimens were similar in all patients with LEMS-SCLC (carboplatin/cisplatin and etoposide median 4 cycles). Four patients (28.6%) received thoracic radiotherapy. Nine patients exhibited complete and partial resolution in LEMS symptoms after chemotherapy or radiation therapy. Two patients had received intravenous immunoglobulin (IVIg, 20 mg per day for 5–7 days) with significant improvement in neurologic symptoms. Death occurred in 8 patients. No patients died as a result of their neurologic symptoms. The median survival of patients is 18 months.

## 4. Discussion

LEMS may occur as a paraneoplastic disorder, most commonly in association with lung cancer. SCLC was predominant histological type [1–10]. LEMS with other types of lung tumors, including adenocarcinoma, large cell neuroendocrine carcinoma, and squamous cell carcinoma, is highly rare [1–10]. Lung adenocarcinoma accompanying LEMS is extremely rare. There are only a few reported cases worldwide [10]. Symptoms of LEMS appeared prior to symptoms of lung cancer in the majority of patients [1]. Diagnostic time of lung cancer was earlier than that of LEMS in the minority of patients. The understanding of LEMS combined with lung cancer was insufficient, the misdiagnosis and delay diagnosis rate was very high, so the early diagnosis is very important. Therefore, once the LEMS is diagnosed, it is necessary to screen for malignant neoplasm, especially lung cancer (for example, using chest CT or tumor markers: neuron-specific enolase and progastrin-releasing peptide, even bronchoscopy) every 6 months for two consecutive years [11]. The role of positron emission tomography (PET-CT) in detecting lung cancer among patients with LEMS remains undetermined. In our study, PET-CT did not serve as the diagnostic clue or measure. Age at onset, smoking history, bulbar involvement, Karnofsky performance status, weight loss, and male impotence were independent predictors for SCLC among LEMS patients [12]. The value of the validated DutchEnglish LEMS Tumor Association Prediction (DELTA-P) score in prediction of the presence of SCLC in LEMS patients had not been confirmed in Chinese population including our series. LEMS was often misdiagnosed as other neuromuscular diseases. Several patients in our study were diagnosed with lung cancer in advanced or extensive stage due to delay diagnosis. We should take a detailed clinical history and perform thorough physical examination and medical instrument examination. The male predominance and advanced age at onset in subjects coexisting with lung cancer and LEMS probably mirrored the characteristics of patients with SCLC, which were similar to previous studies [6, 7]. The clinical course was generally insidious and progressive.

The establishment of LEMS diagnosis mainly depends on clinical manifestation, VGCC antibody, and electrophysiological performance. The symptoms associated with LEMS are due to inhibition in the transmission of the signal mediated by acetylcholine from the presynaptic nerve to skeletal muscles, resulting in muscle weakness. Rare studies reported respiratory muscle involvement in LEMS. LEMS is usually underdiagnosed in patients with respiratory failure of undetermined cause [13, 14]. Previous studies showed that severity of respiratory muscle involvement in such patients is usually mild, with an unspecific restrictive pattern. However, our study reported the largest number of cases with lung cancer coexisting with LEMS developed severe postoperative hypoxemia. Patients with underdiagnosed or untreated LEMS have increased sensitivity to neuromuscular blocking drugs, and therefore, they were high risk group that developed postoperative respiratory failure. Hence, lung function and oxygenation should be evaluated among patients with lung cancer especially during the perioperative period. Given the association of LEMS with lung cancer, the presence of unexplained dyspnea should arise serious suspicion of respiratory muscle weakness due to LEMS.

Muscle weakness commonly spread proximally to distally and caudally to cranially and finally reach the oculobulbar region. The proximal limbs are more commonly affected than the distal aspects. Lower limb weakness accompanied by the decrease or loss of tendon reflex was easily misdiagnosed as symptoms of peripheral neuropathy disease, especially the patients with diabetes mellitus. The clinical suspicion of LEMS is strengthened by concomitant signs of decreased or absent tendon reflexes. Transient increase of the muscle strength and tendon reflexes after short exercise was observed in 40% of LEMS patients. Postexercise facilitation has sound electrophysiological explanation. Therefore, myodynamic examination and tendon reflexes in patients with the suspicion of LEMS should be tested after a short rest period to avoid false negative response [15]. Small number of patients in our study had symptoms of drooping eyelids, double vision, difficulty swallowing, and dysarthria. Unlike myasthenia gravis, isolated extraocular muscle involvement is not common. Several studies revealed half of patients with LEMS exhibited autonomic dysfunction that provided another diagnosis clue [1]. Symptoms or signs of autonomic dysfunction have been found in most of LEMS patients, preceding muscle weakness onset by years. The symptoms of autonomic dysfunction are diverse including dry mouth, constipation, erectile dysfunction, and orthostatic hypotension. Dry mouth is the most common symptom in our study, followed by constipation and male impotence. Dysautonomic symptoms were common in the elderly and lack specificity, which always cannot indicate the diagnosis. The VGCC antibody test has not been widely used in China, and its sensitivity is around 80–90%. Repetitive nerve stimulation (RNS) tests should be performed on at least two distal muscles. The general electromyography characteristics of LEMS was a reduction in action potential amplitude after repetitive peripheral never stimulation at low frequency and increased amplitude at high frequency. Substantial decrease of compound muscle action potential (CMAP) amplitude (decrement) of more than 10% at low stimulating frequencies occurred in all patients in our study. An increase in the CMAP amplitude (increment) of at least 100% are considered to have high specific for the diagnosis of LEMS. Its sensitivity ranged between 84 and 96% [1–17]. The degree of abnormality in CMAP amplitude parallel with the severity of neuromuscular block.

LEMS may be a favorable factor for the prognosis of lung cancer, probably due to early identification of lung cancer and anti-VGCC antibodies that plays an important role in inhibiting tumor growth [18]. Prolonged survival is also observed in patients with LEMS-SCLC whose tumor is extensive at initial diagnosis. The potassium-channel blocker 3,4-diaminopyridine (3,4-DAP) has been previously used for the symptomatic treatment of LEMS [19]. 3,4-DAP is an orphan drug not easily available in China. A single crossover trial reported IVIg significantly improves myometric limb strength [20]. However, till now there is not sufficient data to support the role of IVIg in treatment of lung cancer-associated LEMS. Our institution experience was that IVIg was applied in acute phase to neutralize antibody for 5–7 days. Sakaguchi et al. reported an extensive stage SCLC patient complicated with LEMS successfully treated by immune checkpoint inhibitor plus chemotherapy without a flare-up of LEMS [21].

Several limitations of this study should be acknowledged. First, this study was retrospective in design, and the selection bias and limited statistical power should be considered. Part of patients' records have no validated or uniform measure. Second, respiratory muscle weakness was evaluated based on clinical observation and arterial blood gas measurements in the current study. Phrenic nerve conduction, RNS of the phrenic nerve and needle EMG of the diaphragm tests was not conducted in our centers. Third, there is too small number of participants to conduct full multivariate analysis to eliminate bias from prognostic factors. A large prospective study should be encouraged to further explore the feature of the disease and to explore effective therapies.

## 5. Conclusions

LEMS is an autoimmune disease that frequently occurs in patients with lung cancer.

Although LEMS in lung cancer is relatively rare, early identification of patients coexisting with LEMS and lung cancer is crucial to improving the prognosis of both conditions. Lower extremity weakness accompanying with respiratory symptoms should raise serious suspicion of lung cancer coexisting with LECM. Patients with suspicion of such diseases should be examined and treated by multidisciplinary team including respiratory, neurology, oncology, thoracic, pathology, and radiology department. Considerable research should be further launched to determine the pathophysiological mechanisms in LEMS in lung cancer.

## Figures and Tables

**Table 1:** Demographics of 14 LEMS patients with lung cancer.

Characteristic	No. of patients (%)
Total number	14
Male/female	9/5
Age (years old)	67.1 ± 8.4
Smoking history	10/14
SCLC	13 (92.9%)
Adenocarcinoma	1 (7.1%)
Stage III-IV at diagnosis	9 (64.3%)
Performance status score 0-1	9 (64.3%)
Karnofsky performance score ＞70	9 (64.3%)
Misdiagnosis	12 (85.7%)
Concurrent immunological disorder	3 (21.4%)
Median time between diagnosis of LEMS and detection of the SCLC (months)	5.2 ± 5.5
Median interval between onset of symptoms and completely diagnosis of lung cancer coexisting with LEMS (months)	11.9 ± 7.0

**Table 2:** The symptoms and signs of 14 LEMS patients with lung cancer.

Symptoms	No. of patients (%)
Onset	
Gradual	11 (78.6%)
Acute	3 (21.4%)
Respiratory symptoms and/or signs	8 (57.1%)
Muscle weakness	13 (92.9%)
Leg weakness	13 (92.9%)
Proximal	13 (92.9%)
Distal	7 (50.0%)
Upper extremity weakness	4 (28.6%)
Proximal	4 (28.6%)
Distal	2 (14.3%)
Respiratory muscle weakness	3 (21.4%)
Cranial nerve weakness	5 (35.7%)
Ocular muscle weakness	3 (21.4%)
Oropharyngeal symptoms	4 (28.6%)
Autonomic dysfunction	10 (71.4%)
Dry mouth	8 (57.1%)
Dry eyes	3 (21.4%)
Constipation	6 (42.9%)
Male impotence	2 (14.3%)
Orthostatic hypotension	2 (14.3%)
Decreased or absent tendon reflexes	7 (50.0%)
Restrictive ventilatory dysfunction	3 (21.4%)

## Data Availability

The datasets used and analyzed during the current study are available from the corresponding author on reasonable request.
